The article "Application of Quantitative Assessment Strategy-Based Nursing Combined with Empathic Nursing in Patients Undergoing Tension-Free Inguinal Herniorrhaphy" was retracted in 2023. Reasons: signs of a paper mill; suspected computer-generated content; unreliable results or conclusions; lack of ethics approval or compliance.

# Application of Quantitative Assessment Strategy-Based Nursing Combined with Empathic Nursing in Patients Undergoing Tension-Free Inguinal Herniorrhaphy

**DOI:** 10.1155/2022/7897027

**Published:** 2022-09-29

**Authors:** Yamei Xiang, Lingyun Xi

**Affiliations:** Operation Room, Xi'an No. 1 Hospital (The First Affiliated Hospital of Northwest University), Xi'an 710002, Shaanxi, China

## Abstract

**Objective:**

This study aimed to explore the application of quantitative assessment strategy-based nursing combined with empathic nursing in patients undergoing tension-free inguinal herniorrhaphy.

**Methods:**

82 patients who underwent tension-free inguinal herniorrhaphy in our hospital from May 2020 to December 2021 were enrolled. According to the random number table method, they were divided into three groups (A, B, and C). Patients in group A received quantitative assessment strategy-based nursing combined with empathic nursing, and group B received quantitative assessment strategy-based nursing. Group C received a routine intervention. The early recovery of the three groups was observed. Heart rate (HR), oxygen saturation (SpO_2_), and blood pressure (BP) were recorded before entering the operating room and at the beginning of anesthesia. Mental Health Continuum-Short Form (MHC-SF, adult version) was used to assess the psychological status. The Modified Barthel Index (MBI) score of three groups at different time points was recorded. The complications of the three groups were observed.

**Results:**

Compared with group C, wound healing time, ambulation time, hospital stay time, and time to resume daily activities in groups A and B were significantly shorter (all *P* < 0.05). At the beginning of anesthesia, HR and BP levels in the three groups were all decreased, with HR and BP levels in group A lower than those in group C and HR levels in group B lower than those in group C (all *P* < 0.05). After the intervention, the scores of emotional well-being, psychological well-being, and social well-being in groups A and B were higher than those in group C and the scores of psychological well-being and social well-being in group A were higher than those in group B (all *P* < 0.05). The daily living ability score of group A was higher than that of groups B and group C at discharge, one month after discharge, and three months after discharge, and the daily living ability score of group B was higher than that of group C at these three time points (all *P* < 0.05). No significant differences were observed in the incidence of complication rate among the three groups (10.71%, 14.81%, and 29.63%) (*χ*^2^ = 3.616, all *P* > 0.05).

**Conclusion:**

Quantitative evaluation strategy-based nursing combined with empathic nursing can effectively improve the early recovery of patients undergoing tension-free inguinal herniorrhaphy, reduce their stress response, and improve their mental health and daily living ability.

The article "Application of Quantitative Assessment Strategy-Based Nursing Combined with Empathic Nursing in Patients Undergoing Tension-Free Inguinal Herniorrhaphy" was retracted in 2023. Reasons: signs of a paper mill; suspected computer-generated content; unreliable results or conclusions; lack of ethics approval or compliance.

## 1. Introduction

Inguinal hernia is a common surgical disease. This is associated with increased abdominal muscle strength, which is more common in middle-aged and older adults. The possibility of self-healing of this disease is low, and artificial repair is usually needed. In the face of the operating room environment, patients undergoing tension-free inguinal herniorrhaphy tend to be nervous, which causes a stress response in the body. The sympathetic nerves of patients will be excited, leading to the enhancement of adrenal cortex function [1–3]. Patients with severe stress may have multiple system dysfunction, affecting anesthesia and surgery's smooth operation [4, 5]. Therefore, postoperative intervention for patients undergoing tension-free inguinal herniorrhaphy is critical. Conventional nursing is prone to ignore various emergencies and individual characteristics of patients, showing unsatisfactory nursing effects. Nursing based on a quantitative assessment strategy is a nursing model that carries out comprehensive assessment based on patients' disease risk and then provides targeted nursing. The quantitative evaluation strategy is a widely used nursing model for postoperative rehabilitation patients. Implementing nursing measures based on quantitative and precise evaluation results can make the nursing content more accurate and targeted. This nursing method has been widely applied in clinical practice with remarkable effects, but its application in patients undergoing tension-free inguinal herniorrhaphy remains insufficient [6–8]. Empathy nursing aims to express the understanding of patients' inner changes so that patients can enjoy private nursing services and improve confidence, which will promote the improvement of patients' lousy mood, enable patients to accept surgery with a good attitude, and further promote the smooth operation of the surgery [9, 10]. In the present study, nursing based on a quantitative evaluation strategy combined with empathic nursing was applied to patients with tension-free inguinal herniorrhaphy and the nursing effect was investigated. The results of this study are reported as follows.

## 2. Materials and Methods

### 2.1. General Data

A total of 82 patients undergoing tension-free inguinal herniorrhaphy in our hospital from May 2020 to December 2021 were enrolled, and they were divided into three groups: group A (28 cases), group B (27 cases), and group C (27 cases) according to the random number table method. In group A, there were 18 males and 10 females. The age ranged from 52 to 75 years, with an average of 67.25 ± 7.01 years. Hernia types were found as oblique hernia in 17 cases and direct hernia in 11 cases. Surgical methods included tension-free inguinal hernia repair in 26 cases and laparoscopic inguinal hernia repair in 2 cases. In terms of marital status, there were 22 married cases and 6 single cases (divorced, widowed, and unmarried). Education level was identified as follows: 16 cases of junior middle school or below and 12 cases of senior high school or technical secondary school or above. In group B, there were 20 males and 7 females. The age ranged from 57 to 76 years, with an average of 67.04 ± 5.67 years. Hernia types were found as oblique hernia in 16 cases and direct hernia in 11 cases. Surgical methods included tension-free inguinal hernia repair in 25 cases and laparoscopic inguinal hernia repair in 2 cases. In terms of marital status, there were 18 married cases and 9 single cases (divorced, widowed, and unmarried). Education level was identified as follows: 21 cases of junior middle school or below and 6 cases of senior high school or technical secondary school or above. In group C, there were 16 males and 11 females. The age ranged from 55 to 75 years, with an average of 66.89 ± 6.57 years. Hernia types were found as oblique hernia in 18 cases and direct hernia in 9 cases. Surgical methods included tension-free inguinal hernia repair in 25 cases and laparoscopic inguinal hernia repair in 2 cases. In terms of marital status, there were 24 married cases and 3 single cases (divorced, widowed, and unmarried). Education level was identified as follows: 14 cases of junior middle school or below and 13 cases of high school or technical secondary school or above. The general data of the three groups were comparable (all *P* > 0.05). This study was approved by the hospital ethics committee. Inclusion criteria were as follows: (1) age ≥18 years; (2) all patients diagnosed with an indirect or direct inguinal hernia for the first time; (3) all patients confirmed by imaging examination; (4) patients who underwent tension-free hernia repair; (5) patients with no contraindications; (6) all patients who participated in this study voluntarily. Exclusion criteria were as follows: (1) patients with severe organ dysfunction; (2) patients with an incisional hernia, incarcerated hernia, and strangulated hernia; (3) patients with intestinal perforation and intestinal obstruction; (4) patients with coagulopathy; (5) patients with the disorder of consciousness.

The article "Application of Quantitative Assessment Strategy-Based Nursing Combined with Empathic Nursing in Patients Undergoing Tension-Free Inguinal Herniorrhaphy" was retracted in 2023. Reasons: signs of a paper mill; suspected computer-generated content; unreliable results or conclusions; lack of ethics approval or compliance.

### 2.2. Methods

Group C received the routine nursing intervention, group B received nursing based on quantitative assessment strategy, and group A received nursing based on quantitative assessment strategy combined with empathic nursing intervention.

#### 2.2.1. Group C

Group C received routine nursing and discharge guidance. Patients were urged to refrain from strenuous exercise and return to the outpatient clinic for regular review. In addition, home diet guidance was provided.

#### 2.2.2. Group B

Group B received nursing based on quantitative assessment strategies. (1) A nursing intervention group was established, and a quantitative assessment was developed. A visual analog scale (VAS) [11] was used to evaluate the pain degree of the two groups, and a self-rating anxiety scale (SAS) [12] was used to evaluate the anxiety of the two groups. The total quantified score was calculated according to the quantitative assessment form. Scores >12 were classified as high risk, 9–12 as medium risk, and <9 as low risk. If a single item in the patient quantitative assessment table was ≥2, this item needed to be focused on intervention. (2) The human nursing resources were reasonably allocated. According to the quantitative assessment form score, patients were assigned different numbers of nurses with different grades. Low-risk patients were cared for by 1 nurse with grade NI, medium-risk patients were cared for by 1 nurse with grade N2; high-risk patients were cared for by 1 nurse with grade N3. (3) Nursing table design based on the quantitative assessment strategy is shown in Tables 1 and 2.

#### 2.2.3. Group A

Group A received intervention based on a quantitative assessment strategy combined with empathic nursing. The intervention based on a quantitative assessment strategy was the same as group B, and the empathic nursing was as follows: (1) Establishing an empathic nursing group. The group members should actively understand the relevant content of empathic nursing and carry out nursing interventions after being trained and qualified. (2) Creating a warm operating room atmosphere. Itinerant nurses would reduce the sound of operation nursing operations and walking back and forth, adjust the audio and tone status of the device alarm sound within an appropriate range, play soft music, and reduce the anxiety, helplessness, and loneliness of patients. If patients do not like listening to music, they can turn off the music according to their needs of patients. (3) Eye contact and body communication. A comfortable position was chosen for the patient, and gentle and skilled nursing actions were adopted. In this process, we can strengthen eye contact with patients, keep them warm, hold their hands, comfort and encourage them, and convey the information of care and encouragement.

The article "Application of Quantitative Assessment Strategy-Based Nursing Combined with Empathic Nursing in Patients Undergoing Tension-Free Inguinal Herniorrhaphy" was retracted in 2023. Reasons: signs of a paper mill; suspected computer-generated content; unreliable results or conclusions; lack of ethics approval or compliance.

### 2.3. Observation Targets

(1) Early recovery, (2) stress response, heart rate (HR), oxygen saturation (SpO_2_), and blood pressure (BP) in the three groups were recorded before entering the operating room and at the beginning of anesthesia. (3) Mental health level. The level of positive mental health was assessed by using the Mental Health Continuum-Short Form (MHC-SF, adult version) [13], which consists of 14 items, including mood (3 items) (0∼15 points), psychology (6 items) (0∼30 points), and social well-being (5 items) (0∼25 points). Based on the range of “never∼every day (0∼5 points),” the higher the score, the better the patient's psychological condition. (4) Ability of daily living (ADL) at different time points. The ADL of the three patient groups was assessed using the Chinese version of the Modified Barthel Index (MBI) scale [14]. The scale included 8 self-care activities of eating, toilet, bathing, dressing, transferring, and urine control and 2 behavior-related activities of walking or wheelchair walking for 50 m and going up and down stairs. The total score was 100 points. The higher the score, the better the independence. (5) Incidence of complications.

### 2.4. Statistical Approach

An SPSS 20.0 statistical software was used to analyze and process the data. Measurement data were expressed as ($\bar{x}$ ± *S*). An independent sample *t*-test was used for intergroup comparison, and paired *t*-test was used for intragroup comparison before and after the intervention. Counting data were expressed as frequency and constituent ratio and subjected to the *χ*^2^ test. *P* < 0.05 indicated that the difference was statistically significant.

## 3. Results

### 3.1. Comparison of Early Recovery among Three Groups

The wound healing time, ambulation time, hospital stay time, and time to resume daily activities in groups A and B were significantly shorter than in group C (*P* < 0.05, Table 3).

### 3.2. Comparison of Stress Response of Three Groups before and after Intervention

When entering the operating room, there were no significant differences in HR, SpO_2_, and BP levels among the three groups (all *P* < 0.05). At the beginning of anesthesia, the HR and BP levels in the three groups were decreased; moreover, the HR and BP levels in group A were lower than those in group C, and HR level in group B was lower than that in group C, with statistically significant differences (all *P* < 0.05, Table 4).

### 3.3. Comparison of Positive Mental Health among Three Groups

Before the intervention, there were no significant differences in emotional, psychological, and social well-being scores among the three groups (all *P* > 0.05). After the intervention, the scores of emotional well-being, psychological well-being, and social well-being in groups A and B were higher than those in group C, the scores of psychological well-being and social well-being in group A were higher than those in group B, and the differences were statistically significant (all *P* < 0.05, Table 5).

The article "Application of Quantitative Assessment Strategy-Based Nursing Combined with Empathic Nursing in Patients Undergoing Tension-Free Inguinal Herniorrhaphy" was retracted in 2023. Reasons: signs of a paper mill; suspected computer-generated content; unreliable results or conclusions; lack of ethics approval or compliance.

### 3.4. Comparison of ADL among Three Groups at Different Time Points

The ADL score of group A was higher than that of group B and group C at discharge, 1 month after discharge, and 3 months after discharge, and the ADL score of group B was higher than that of group C at these three-time points (all *P* < 0.05, Table 6).

### 3.5. Comparison of Complications among the Three Groups

There were no significant differences in the incidence of complications among the three groups (10.71%, 14.81%, and 29.63%) (*χ*^2^ = 3.616, *P* > 0.05, Table 7).

## 4. Discussion

Inguinal hernia is a common and frequently occurring disease in clinics, which is easy to recur. Clinically, it is believed that the crucial causes of the disease are mainly the decrease in abdominal wall strength and the increase in intra-abdominal pressure [15]. At present, the clinical treatment of inguinal hernia is mainly surgery. Tension-free hernia repair is widely used because of its low recurrence rate, light pain, fast recovery time, etc. [16]. It has a pronounced therapeutic effect on inguinal hernia patients and puts forward higher requirements for nursing. In addition, it is worth noting that surgery is a traumatic stress response, and postoperative pain is an inevitable, normal physiological response, which will cause patients to have physiological and psychological abnormal reactions, which may affect the curative effect of surgery [17]. Therefore, in addition to the effective surgical treatment of inguinal hernia patients, we should comprehensively consider patients' physical and mental symptoms and implement targeted nursing interventions, to provide more references for improving the overall surgical efficacy and quality of life of patients. However, the effect of conventional operating room nursing is not satisfying. Conventional psychological intervention through the psychological communication and counseling of patients, but the occurrence and prognosis of the disease lack attention, and the psychological problems and coping styles of patients are insufficient. The application of routine psychological intervention in patients with hernia repair has certain limitations. Quantitative assessment is a prospective nursing method. After a comprehensive evaluation of the patient's gender, age, education level, pain, and severity of the condition, the patients are divided into different levels of nursing subjects. When taking intervention for patients, different levels of intervention nursing should be given to each level subject to implementing stratified personalized nursing [18, 19]. According to relevant studies, implementing stratified nursing after comprehensive evaluation can effectively promote patient rehabilitation and reduce the length of hospital stay. Quantitative assessment can clear individual nursing risks, strengthen nursing intensity for high-risk patients, and do an excellent job in every nursing step. Empathy nursing refers to the utmost care given to patients during the smooth operation of nursing. Nurses should consider patients' perspectives and meet their physiological and psychological needs to the maximum [20, 21].

The article "Application of Quantitative Assessment Strategy-Based Nursing Combined with Empathic Nursing in Patients Undergoing Tension-Free Inguinal Herniorrhaphy" was retracted in 2023. Reasons: signs of a paper mill; suspected computer-generated content; unreliable results or conclusions; lack of ethics approval or compliance.

In the present study, 28 patients undergoing tension-free inguinal herniorrhaphy were given nursing based on a quantitative evaluation strategy combined with empathic nursing. After intervention, group A (nursing based on quantitative assessment strategy combined with empathic nursing) and group B (nursing based on quantitative assessment strategy) had significantly shorter wound healing time, time to get out of bed, length of hospital stays, and time to resume daily activities compared with group C (conventional nursing). This indicates that nursing based on a quantitative evaluation strategy combined with empathic nursing can effectively improve the postoperative recovery of patients undergoing tension-free inguinal herniorrhaphy. Nurses should consider patients' perspectives and meet their physiological and psychological needs to the maximum extent. These data can help nurses understand the primary physiological conditions of patients and make the risks of surgery clearer so that nursing staff can make a targeted nursing intervention for surgical risk and ultimately promote postoperative recovery of patients.

Empathy nursing encouraged and comforted patients through language and body, established the confidence of patients to overcome the disease, improved their psychological comfort, and reduced their stress response. Therefore, at the beginning of anesthesia, HR and BP levels in the three groups were decreased; HR and BP in group A were lower than that in group C, and HR in group B was lower than that in group C, all with statistically significant differences (all *P* < 0.05). With the approaching operation time, the patient may appear apparent anxiety state before surgery, and the patient's physiological stress response is strengthened. What is worse, patients' excessive anxiety and fear can trigger the secretion of substances such as norepinephrine and adrenaline, activate the sympathetic adrenal medulla system, and increase nerve excitability, resulting in vasoconstriction, shortness of breath, and increased blood pressure, affecting the safety of surgery [22, 23].

The article "Application of Quantitative Assessment Strategy-Based Nursing Combined with Empathic Nursing in Patients Undergoing Tension-Free Inguinal Herniorrhaphy" was retracted in 2023. Reasons: signs of a paper mill; suspected computer-generated content; unreliable results or conclusions; lack of ethics approval or compliance.

Based on the quantitative assessment strategy, the nurse deepened the nurse-patient relationship during the communication of essential information with patients, and the psychological pressure of patients was relieved to a certain extent. Therefore, the improvement of stress response in group B was better than in Group C, and the patients in group A given empathic nursing further improved their stress response. After the intervention, the scores of emotional well-being, psychological well-being, and social well-being in groups A and B were higher than those in group C and the scores of psychological well-being and social well-being in group A were higher than those in group B, with statistical significances (all *P* < 0.05). This showed that quantitative assessment strategy-based nursing combined with empathy nursing had the best results in improving the positive health level of patients, followed by nursing intervention based on the strategy of quantitative assessment alone. This may be because the interventions based on quantitative assessment strategies and empathic nursing enhanced patient-nurse communication. Patients and their families were more willing to cooperate; their psychological pressure was smaller. Moreover, nursing based on a quantitative assessment strategy promotes the postoperative recovery of patients. This method carried out targeted pain and psychological intervention for patients. Hence, the positive mental health level of group A and group B was superior to group C. Group A combined with empathy nursing further improved the mental health of patients, so the improvement of positive mental health level in group A was better than that in group B. The ADL scores of group A at discharge, 1 month after discharge, and 3 months after discharge were higher than those of groups B and C, and the ADL score of group B at discharge, 1 month after discharge, and 3 months after discharge was higher than that of group C (all *P* < 0.05). It is suggested that the patients with combined intervention had the best recovery and the intervention based on a quantitative assessment strategy combined with empathy nursing can promote the recovery of patients more effectively. There was no significant difference in complications among the three groups, indicating that nursing based on quantitative assessment strategy and empathic nursing could not improve complications.

The article "Application of Quantitative Assessment Strategy-Based Nursing Combined with Empathic Nursing in Patients Undergoing Tension-Free Inguinal Herniorrhaphy" was retracted in 2023. Reasons: signs of a paper mill; suspected computer-generated content; unreliable results or conclusions; lack of ethics approval or compliance.

In conclusion, intervention based on a quantitative evaluation strategy combined with empathic nursing can improve postoperative recovery, stress response, positive mental health level, and ADL of patients undergoing tension-free inguinal herniorrhaphy, showing clinical application value.

## Figures and Tables

**Table 1:** Quantitative assessment form.

Item	1 point	2 points	3 points
Age			
Pain degree	≤3 points	4∼6 points	7∼10 points
Anxiety	Mild	Moderate	Severe
Complications of cardiovascular disease	No	1	≥2
Educational level	College degree or above	Senior high school/technical secondary school	Junior high school

**Table 2:** Nursing table based on the quantitative evaluation strategy.

Item	Intervention content	Specific operation
Psychological intervention	Establish a good nurse-patient relationship, listen to the patients' preoperative feelings, dredge the patients' destructive emotions, divert the patients' attention through TV, music, books, and other ways, and give the patients' family members corresponding care guidance.	The intervention time of low-risk patients was 30∼40 min/d, that of medium-risk patients was 50∼60 min/d, and that of high-risk patients was 60∼80 min/d.

Health education	Each patient was given a health manual. Before the operation, a wardmate exchange meeting was held and a centralized education was conducted. Individual education and guidance were carried out to explain the precautions for postoperative recovery.	Low-risk patients were given individual education and guidance once, medium-risk patients were given individualized education guidance twice, and high-risk patients were given individualized education guidance three times before operation.

Pain care	Posture intervention and individualized analgesia were performed after the operation.	The patients were given individualized analgesia after the operation. Patients with ≤5 points were given analgesic nursing methods; patients with ≥6 points were given analgesic nursing methods along with drug analgesia according to the doctor's advice. The patients at intermediate and high risk were given distraction interventions, such as playing slow music and chatting with patients.

Early postoperative functional exercise	Carry out early functional exercise in different periods and stages.	(1) 2∼6 h after the operation, the nursing staff massaged the muscles of both the patient's lower limbs, from top to bottom, from the outside to the inside. The massage time for each side was 4∼5 min. After the massage of the lower limbs, the patient performed passive movement of the foot and ankle joints to move gently and slowly, 5∼10 times for each group, two groups a day. After the exercise, the patient turned over once. (2) 6∼12 h after operation, the patients were instructed to perform voluntary contraction of upper and lower limbs and trunk muscles and to perform muscle exercises, including biceps brachii, quadriceps femoris, respiratory muscle, and gastrocnemius muscle. Patients were instructed to perform exercises such as over flexion and overextension of the dorsum of the foot and internal and external rotation of the ankle joint, 10–15 times in each group, 3 groups per day. (3) 12∼24 h after operation, the patients were instructed to perform leg lifting, knee extension and flexion, hip adduction and abduction, shoulder adduction and abduction, elbow extension and flexion, arms lifting, and other exercises, 10∼15 times per group, 3 groups per day. (4) 24∼48 hours after the operation, the patient turned over once every 2 hours under the guidance of the nurse and performed bed sitting and standing training, 3∼5 min each time, 3 times a day, standing and sitting beside the bed, 3∼5 min each time, 2 times a day. (5) 48∼72 hours after the operation, the patients were assisted in getting out of bed activities, 500∼800 steps a day, and the patients were guided to perform simple daily activities. (6) 72 h after the operation, walking exercise was performed with the aid of a walker according to the recovery condition of the patients.

Continuous intervention after discharge	After discharge, formulate a family nursing intervention plan for patients.	A family continuity nursing plan was performed for the patients two days before discharge. The nursing staff in the family were trained to express their concern for the elderly patients from the psychological and daily life aspects. The medical staff conducted a telephone follow-up every two weeks. The following content included the patient's diet, exercise, and medication. A rehabilitation plan was made for the patients according to their situation, and the patients were urged to follow the doctor's advice. The patient shall have a regular blood routine and liver and kidney function examinations, and the attending doctor shall be informed of any abnormalities. The patient's family members were informed to keep the room clean and tidy, change the bed sheets regularly, and ensure room ventilation.

The article "Application of Quantitative Assessment Strategy-Based Nursing Combined with Empathic Nursing in Patients Undergoing Tension-Free Inguinal Herniorrhaphy" was retracted in 2023. Reasons: signs of a paper mill; suspected computer-generated content; unreliable results or conclusions; lack of ethics approval or compliance.

**Table 3:** Comparison of early recovery among three groups ($\bar{x}$ ± *s*).

Group	Wound healing time (h)	Ambulation time (h)	Hospital stay time (h)	Time to resume daily activities (d)
Group A (*n* = 28)	24.14 ± 3.66^②③^	12.93 ± 3.56^②③^	94.96 ± 8.85^②③^	2.36 ± 0.49^②③^
Group B (*n* = 27)	28.04 ± 2.79^②^	20.19 ± 2.60^②^	125.22 ± 12.53^②^	3.48 ± 0.70^②^
Group C (*n* = 27)	30.15 ± 3.73^③^	35.96 ± 3.17^③^	157.33 ± 15.37^③^	4.33 ± 0.48^③^

*Note.* Compared with group C, ^②^*P* < 0.05; with group B, ^③^*P* < 0.05.

**Table 4:** Comparison of stress response of three groups before and after intervention ($\bar{x}$ ± *s*).

Group		Group A (*n* = 28)	Group B (*n* = 27)	Group C (*n* = 27)
HR (time/min)	When entering the operating room	85.70 ± 8.00	84.67 ± 7.88	85.93 ± 6.33
	At the beginning of anesthesia	70.64 ± 5.27^①②③^	75.16 ± 6.18^①②^	80.15 ± 5.89^①③^

SpO_2_ (%)	When entering the operating room	97.40 ± 7.42	98.01 ± 9.34	97.18 ± 9.63
	At the beginning of anesthesia	96.51 ± 9.45	96.88 ± 10.77	96.70 ± 10.54

DBP (mmHg)	When entering the operating room	80.37 ± 5.64	80.63 ± 4.85	80.57 ± 5.21
	At the beginning of anesthesia	72.44 ± 5.76^①②③^	76.15 ± 4.36^①②^	78.05 ± 6.12^①③^

SBP (mmHg)	When entering the operating room	121.74 ± 6.17	121.98 ± 5.81	121.66 ± 7.31
	At the beginning of anesthesia	114.51 ± 5.28^①②③^	116.45 ± 6.41^①②^	118.62 ± 5.33^①③^

*Note.* HR: heart rate; DBP: diastolic blood pressure; SBP: dystolic blood pressure. Compared with the time entering the operation room, ^①^*P* < 0.05; with group C, ^②^*P* < 0.05; with group B, ^③^*P* < 0.05.

**Table 5:** Comparison of positive mental health among three groups ($\bar{x}$ ± *s*).

Group	Emotional well-being		Psychological well-being		Social well-being	
	Before intervention	After intervention	Before intervention	After intervention	Before intervention	After intervention
Group a (*n* = 28)	9.79 ± 1.97	13.43 ± 0.88^①②^	20.07 ± 3.79	27.25 ± 1.73^①②③^	15.18 ± 2.52	21.68 ± 3.08^①②③^
Group B (*n* = 27)	9.11 ± 2.19	12.67 ± 2.09^①②^	20.96 ± 3.74	26.37 ± 2.37^①②^	15.00 ± 1.66	19.48 ± 3.40^①②^
Group C (*n* = 27)	9.07 ± 2.09	10.85 ± 1.73^①③^	20.11 ± 3.29	24.30 ± 2.73^①③^	14.96 ± 1.48	17.81 ± 1.80^①③^

*Note.* Compared with before intervention, ^①^*P* < 0.05; with group C, ^②^*P* < 0.05; with group B, ^③^*P* < 0.05.

**Table 6:** Comparison of ADL among three groups at different time points ($\bar{x}$ ± *s*).

Group	At discharge	1 month after discharge	3 months after discharge
Group a (*n* = 28)	70.86 ± 5.39^②③^	76.11 ± 5.31^①②③^	84.71 ± 7.08^①②③^
Group B (*n* = 27)	64.22 ± 5.39^②^	70.07 ± 6.60^①②^	79.22 ± 5.70^①②^
Group C (*n* = 27)	57.74 ± 5.95^③^	63.22 ± 3.72^①③^	70.52 ± 5.03^①③^

*Note.* Compared with discharge, ^①^*P* < 0.05; with group C, ^②^*P* < 0.05; with group B, ^③^*P* < 0.05.

**Table 7:** Comparison of complications among the three groups (cases (%)).

Group	Recrudescence	Wound infection	Subcutaneous hematoma	Total complication rate
Group A (*n* = 28)	1 (3.57)	1 (3.57)	1 (3.57)	3 (10.71)
Group B (*n* = 27)	1 (3.70)	1 (3.70)	2 (7.41)	4 (14.81)
Group C (*n* = 27)	3 (11.11)	2 (7.41)	3 (11.11)	8 (29.63)

The article "Application of Quantitative Assessment Strategy-Based Nursing Combined with Empathic Nursing in Patients Undergoing Tension-Free Inguinal Herniorrhaphy" was retracted in 2023. Reasons: signs of a paper mill; suspected computer-generated content; unreliable results or conclusions; lack of ethics approval or compliance.

## Data Availability

The labeled dataset used to support the findings of this study is available from the corresponding author upon request.
